The article "The influence of iatrogenic atrial septal defect on the prognosis of patients with atrial fibrillation between cryoablation and radiofrequency ablation" was published in 2020. Journal: Biosci Rep.

# The influence of iatrogenic atrial septal defect on the prognosis of patients with atrial fibrillation between cryoablation and radiofrequency ablation

**DOI:** 10.1042/BSR20193128

**Published:** 2020-02-07

**Authors:** Ying Yang, Jinglan Wu, Lixia Yao, Yue Liu, Chenfeng Zhang, Ling You, Jing Yang, Ruiqin Xie

**Affiliations:** Department of Cardiology, The Second Hospital of Hebei Medical University, Shijiazhuang 050000, China

**Keywords:** atrial fibrillation, cardiac function, cryoablation, iatrogenic atrial septal defect, prognosis, radiofrequency ablation

## Abstract

**Objective:** The present study was to compare the incidence of septal defect (SD) in patients with atrial fibrillation (AF) who received radiofrequency ablation or cryoablation.

**Methods:** A total of 293 AF patients were performed with radiofrequency ablation and cryoablation. Cardiac ultrasonography was performed to calculate left atrial diameter (LAD), left atrial ejection fraction (LAEF%), strain rate (SR), left ventricular systolic (SRs), left ventricular diastolic (SRe), and left atrial systole (SRa) before surgery, 3 months and 1 year after surgery. The patients were followed up to observe statin and angiotensin-converting enzyme inhibitor (ACEI)/angiotensin receptor blocker (ARB) medication, AF recurrence, 6-min walk test, stroke, any symptoms caused by arrhythmia, and re-hospitalization. **Results:** The levels of LAD and SD were higher, while SRe and SRa were lower in the cryoablation group in the comparison with the radiofrequency ablation group after surgery (*P*<0.05). LAEF was lower in the cryoablation group than the radiofrequency ablation group after 3 months (*P*<0.05). After 1-year follow-up, no right-to-left shunt occurred in all patients with SD. The AF recurrence rate in SD group was higher than that in the normal group (*P*<0.05). The use of statin and the application of ACEI/ARB were protective factors, whereas hypertension, LAD, left atrial operation time, and surgical plan were risk factors. **Conclusion:** SD affects left atrial function and increases the risk of AF recurrence. Hypertension, LAD, and left atrial operation time are risk factors for SD, whereas statin and ACEI/ARB drugs can reduce SD.

## Introduction

Pulmonary vein triggered atrial fibrillation (AF) theory makes pulmonary vein isolation (PVI) the basis for the treatment of AF [1]. Under the guidance of this theory, in recent years, PVI has been increasingly used to treat AF with poor drug treatment effect [2]. Initially, this procedure was performed by controlling the ablation catheter to abruptly separate the pulmonary veins through RF energy ‘point by point’. However, the procedure requires high technique, long operation time, and fluoroscopy time, and it brings obvious pain [3]. Subsequently, the frozen balloon technique appeared and developed rapidly. The cryoablation method is easy to learn and master, resulting in shorter learning time [4–5]. So far, there are many clinical trials aiming to prove that cryoablation is safe and effective. There is no significant difference on the short-term and long-term results between radiofrequency ablation and cryoablation isolation of pulmonary veins for AF [6–9]. For these reasons, more and more clinicians choose frozen balloon technology to treat AF. Regardless of the technique used, the first step in PVI ablation is to establish a right to left atrium channel through atrial septal puncture. During follow-up, we found that some patients suffered from persistent septal defect (SD), and its incidence in patients with frozen balloon ablation was significantly higher than that in patients with radiofrequency ablation. Based on this finding, we observed patients under different operations to compare the incidence of SD and explored the risk factors, protective factors, and its clinical significance.

The article "The influence of iatrogenic atrial septal defect on the prognosis of patients with atrial fibrillation between cryoablation and radiofrequency ablation" was published in 2020. Journal: Biosci Rep.

## Materials and methods

### Patients

A total of 293 patients with AF underwent PVI treatment in our center from December 2015 to December 2017 were enrolled. They were divided into two groups according to different catheter ablation methods. There were 152 patients in the radiofrequency ablation group, including 91 males and 61 females with mean age of 57.88 ± 9.83 years (ages ranged from 32 to 76 years). There were 141 patients in the cryoablation group, including 78 males and 63 females with average age of 60.24 ± 10.8 years (ages ranged from 31 to 77 years).

Inclusion criteria: patients with AF underwent catheter ablation, including paroxysmal and persistent AF. Exclusion criteria: patients with (1) severe liver and kidney dysfunction or other systemic diseases; (2) AF caused by rheumatic heart disease, idiopathic cardiomyopathy, coronary heart disease, severe hypertension, or hyperthyroidism; (3) contraindications to radiofrequency ablation; (4) received radiofrequency ablation for AF before; (5) atrial SD.

## Methods

### Operation

The patients received low molecular weight heparin for anticoagulation before operation. All the patients had signed informed consent. Catheter ablation procedure was performed by the same surgeon. Surgical procedure: (1) Cryoablation group: a lead catheter was put into coronary sinus through puncturing left femoral vein, an electrode was placed in superior vena cava through left femoral vein for spare pacing, and the right femoral vein was punctured as a frozen balloon catheter approach. Atrial septal puncture and pulmonary vein computed tomography (CT) combined with CARTO imaging were routinely performed to show pulmonary vein opening and vestibular. A balloon-type cryoablation catheter with achieve ring-shaped electrode (28 or 23 mm, Arctic Front Advance, Medtronic Cryocath LP) was placed through FlexCath Advance controllable long sheath (15F). The achieve electrode was sequentially sent to each pulmonary vein, and the position and direction of the balloon were adjusted to block the opening of the pulmonary vein. After the sealing was good indicated by the angiography, the liquid nitrogen was used for frozen and ablation with the decrease of temperature to the range from −40 to −60°C. The sequence was from the upper left, lower left, and upper right to the lower right pulmonary veins. Each pulmonary vein was frozen 2–6 times, and each time of freezing was shorter than 180 s to electrically isolate the pulmonary vein completely. When the right pulmonary vein was isolated, the superior vena cava continuously paced the phrenic nerve to determine whether the phrenic nerve was damaged or not. (2) Radiofrequency ablation group: the left aortic vein was punctured to deliver the lead catheter into the coronary sinus. The right femoral vein approach was performed to complete the atrial septal puncture (1 time) and a Swartz SL1 long sheath (8.5F) was placed. The left atrium anatomy was constructed under the guidance of the CARTO3 three-dimensional mapping system. The Lasso ring electrode and cold saline navigation pressure ablation catheter were placed for circumferential venous potential vestibular isolation till the pulmonary vein potential completely disappeared. Parallel pacing was performed to confirm the two-way block between the pulmonary vein and the heart chamber.

The article "The influence of iatrogenic atrial septal defect on the prognosis of patients with atrial fibrillation between cryoablation and radiofrequency ablation" was published in 2020. Journal: Biosci Rep.

### Observation index

Medical history, physical examination, laboratory examination, routine electrocardiogram and dynamic electrocardiography, cardiac ultrasonography, and cardiac CT (pulmonary vein and left atrial three-dimensional reconstruction) were performed on patients before treatment. B-type natriuretic peptide (BNP), HR-C-reactive protein (HR-CRP), Troponin I (TNI), and Creatine kinase-MB (CK-MB) were measured in all patients before and 24 h after surgery. All patients underwent cardiac ultrasonography to measure left atrial diameter (LAD) before, 3 months, and 1 year after surgery. Left atrial ejection fraction (LAEF%): The maximum volume of the left atrium at the end of the left ventricle (LAV_max_) and the minimum volume of the left atrial end of the diastolic (LAV_min_) were measured. LAEF% = (LAV_max_ − LAV_min_)/LAV_max_ × 100%. Left atrial strain (S%) and strain rate (SR): left ventricular systolic (SRs), left ventricular diastolic (SRe), left atrial systole (SRa): start CMQ mode, respectively obtain apical two-chamber and four-chamber sections. The maximum volume image of the left atrium was selected, and the sampling points were placed on the septal side, the side wall, and the atrial top of the left atrium to obtain the SR curve of the four chambers. The sampling points were placed on the lower wall, the anterior wall, and the atrial top to obtain the SR curve of the two chambers. All indicators were measured continuously for three cardiac cycles to calculate the average value by experienced sonographer. Atrial ultrasound and left atrial function were observed by cardiac ultrasound two-dimensional speckle tracking.

### Postoperative treatment and follow-up

Routine medication was given after surgery. Low molecular weight heparin was given for 1 to 2 days and then replaced with rivaroxaban 15–20 mg/day, dabigatran capsule 110 mg/day, or oral warfarin to maintain international normalized ratio (INR) value between 2 and 3. Anticoagulant drugs were discontinued after 3 months of oral administration. Statin and angiotensin-converting enzyme inhibitor (ACEI)/angiotensin receptor blocker (ARB) medication, AF recurrence, 6-min walk test, stroke, any symptoms caused by arrhythmia, and re-hospitalization were followed up.

### Statistical analysis

All data analyses were performed using SPSS19.0 statistical software. The measurement data with the normal distribution were expressed as means ± standard deviation $\bar{x}\;\pm \;s$ and compared by *t* test. The enumeration data were expressed as the rate (%) and compared by χ^2^ test. The correlation multivariate analysis was performed by logistic regression analysis. *P*<0.05 was considered to be statistically different.

## Results

Radiofrequency ablation was successfully completed in all patients without pulmonary vein stenosis. There was no thromboembolic event, pericardial tamponade, left atrial rupture, left atrial esophageal fistula, and other complications observed.

### Basic information comparison

There were no statistical differences in age, sex, body mass index (BMI), hypertension, diabetes mellitus, cerebrovascular disease, cardiac insufficiency, basal heart rate, ratio of onset to persistent AF, statin and ACEI/ARB medication, baseline BNP, HR-CRP, TNI, and CKMB between the two groups (*P*>0.05, Table 1). There were no significant differences on the baseline color echocardiography between the two groups (*P*>0.05, Table 2).

**Table 1:** Basic information comparison

Index	CB	RF	T value/χ^2^ value	*P*-value
Age	60.24 ± 10.80	57.88 ± 9.83	1.958	0.051
Gender (male/female)	78/63	91/61	0.620	0.431
BMI	25.62 ± 5.58	26.07 ± 3.51	0.832	0.406
Hypertension (*n*)	84	74	3.492	0.062
Paroxysmal AF (*n*)	69	74	0.002	0.964
Diabetes (*n*)	22	23	0.012	0.912
Cerebrovascular disease (*n*)	23	19	0.87	0.352
Heart dysfunction (*n*)	22	26	0.12	0.728
Heart rate (times/min)	77.77 ± 19.00	82.41 ± 19.84	1.935	0.054
Statins (*n*)	67	71	0.019	0.890
ACEI/ARB (*n*)	56	53	0.736	0.391
BNP	106.63 ± 81.98	107.46 ± 100.95	0.077	0.939
HR-CRP	1.81 ± 1.59	1.86 ± 1.66	0.263	0.793
TNI	0.013 ± 0.008	0.010 ± 0.008	1.425	0.155
CKMB	13.83 ± 4.84	14.08 ± 5.89	0.395	0.693

The article "The influence of iatrogenic atrial septal defect on the prognosis of patients with atrial fibrillation between cryoablation and radiofrequency ablation" was published in 2020. Journal: Biosci Rep.

**Table 2:** Basal ultrasound index comparison

Index	CB	RF	T value/χ^2^ value	*P*-value
LAD	36.32 ± 4.18	37.06 ± 4.77	1.408	0.160
RAD	35.31 ± 4.25	36.20 ± 3.23	1.897	0.059
E peak	71.40 ± 20.21	71.47 ± 18.70	0.028	0.978
A peak	69.71 ± 12.19	71.08 ± 17.55	0.537	0.592
E/A peak	1.09 ± 0.37	1.20 ± 0.45	1.617	0.108
S%	29.23 ± 12.59	29.07 ± 11.79	0.118	0.906
SRs	1.60 ± 0.54	1.50 ± 0.52	1.492	0.137
SRe	−1.81 ± 0.61	−1.89 ± 0.86	0.811	0.418
SRa	−2.37 ± 0.74	−2.24 ± 0.62	1.104	0.271
LAEF	45.07 ± 15.02	45.83 ± 14.77	0.435	0.664
LVEF	61.13 ± 7.60	61.76 ± 8.08	0.684	0.495

## Index comparison

### Atrial SD incidence comparison

At 3 months after operation, most of the interatrial septal punctures were closed. The incidence of atrial SD in the cryoablation group (15F sheath) was significantly higher than that in the radiofrequency ablation group (8.5F sheath) (24.11 vs. 11.84%, *P*<0.05). At 1 year after operation, the incidence of atrial SD in the cryoablation group (15F sheath) was still obviously higher than that in the radiofrequency ablation group (8.5F sheath) (15.60 vs. 6.58%, *P*<0.05). At 1 year of follow-up, no right-to-left shunt occurred in all patients with atrial SD (Table 3).

**Table 3:** Comparison of ASD incidence in two groups at 3 months and 1 year after operation

Index	3 months		*P*-value	1 year		*P*-value
	CB	RF		CB	RF	
Incidence rate (%)	34 (141)	18 (152)	0.006	22 (141)	10 (152)	0.014

### Comparison of ultrasound indexes at 3 months and 1 year after operation

LAD showed no statistical difference at 3 months (*P*>0.05) and was higher in the cryoablation group than that in the radiofrequency ablation group after 1 year (*P*<0.05). There were no significant differences in RAD, E peak, A peak, E/A value, S%, SRs, and LVEF at 3 months and 1 year between the two groups (*P*>0.05). SRe exhibited no statistical difference at 3 months (*P*>0.05) and was lower in the cryoablation group than that in the radiofrequency ablation group after 1 year (*P*<0.05). SRa in the cryoablation group was markedly lower than that in the radiofrequency ablation group at both 3 months and 1 year (*P*<0.05). LAEF showed no statistical difference at 1 year (*P*>0.05), but it was lower in the cryoablation group than that in the radiofrequency ablation group after 3 months (*P*<0.05). The SD incidence in the cryoablation group was significantly higher than that in the radiofrequency ablation group at both 3 months and 1 year (*P*<0.05). At one-year follow-up, no right-to-left shunt occurred in all SD patients (Table 4).

The article "The influence of iatrogenic atrial septal defect on the prognosis of patients with atrial fibrillation between cryoablation and radiofrequency ablation" was published in 2020. Journal: Biosci Rep.

**Table 4:** Iintra- and postoperative indicator comparison

Index	CB	RF	T value/χ^2^ value	*P*-value
BNP	119.29 ± 96.70	108.01 ± 98.94	1.021	0.308
HR-CRP	5.79 ± 2.28	4.52 ± 2.05	5.020	<0.001
TNI	6.06 ± 2.72	1.84 ± 1.08	17.722	<0.001
CKMB	50.10 ± 16.34	22.60 ± 8.64	18.19	<0.001
Exposure time	9.74 ± 3.44	3.51 ± 1.34	19.56	<0.001
Left atrial operation time	74.43 ± 25.44	114.09 ± 28.26	12.27	<0.001
Recurrence (case)	41	51	0.68	0.409

### Comparison of indicators between SD and non-SD groups

The recurrence rate of AF in patients with SD was significantly higher than that in the normal group (53.13 vs.28.74%, *P*<0.05). Subgroup analysis showed that the recurrence rate of AF was markedly higher in patients with IASD than that in patients without IASD in the cryoablation group at 1 year (50.00 vs.27.73%, *P*<0.05). The recurrence rate of AF in patients with IASD was also apparently higher than that in patients without IASD in the radiofrequency ablation group at 1 year (60.00 vs.29.58%, *P*<0.05) (Table 5).

**Table 5:** Echocardiography comparison after operation

Index	3 months		*P*-value	1 year		*P*-value
	CB	RF		CB	RF	
LAD	36.50 ± 3.86	36.01 ± 4.02	0.299	35.87 ± 3.55	35.07 ± 3.31	0.047
RAD	34.57 ± 3.18	35.26 ± 2.83	0.064	34.01 ± 2.92	34.44 ± 2.36	0.189
E peak	73.67 ± 19.84	74.19 ± 18.13	0.68	78.01 ± 19.73	76.68 ± 15.71	0.52
A peak	67.83 ± 14.14	71.43 ± 14.01	0.043	70.95 ± 13.25	73.98 ± 12.35	0.087
E/A value	1.13 ± 0.46	1.10 ± 0.36	0.491	1.14 ± 0.35	1.08 ± 0.30	0.183
S%	30.31 ± 9.72	31.18 ± 9.98	0.471	34.22 ± 8.91	34.53 ± 10.92	0.802
SRs	1.53 ± 0.47	1.57 ± 0.58	0.591	1.73 ± 0.38	1.76 ± 0.49	0.581
SRe	−1.67 ± 0.56	−1.80 ± 0.72	0.104	−1.73 ± 0.56	−1.95 ± 0.81	0.011
SRa	−1.84 ± 0.64	−2.04 ± 0.83	0.031	−2.31 ± 0.63	−2.53 ± 0.75	0.015
LAEF	53.35 ± 11.89	56.54 ± 11.83	0.022	51.81 ± 13.57	54.13 ± 15.37	0.173
LVEF	63.96 ± 6.31	63.61 ± 5.97	0.626	65.66 ± 6.23	66.88 ± 4.45	0.054
SD	34	18	0.006	22	10	0.013

There were no significant differences in LAD, RAD, A peak, SRa, and the use of statin before operation between the two groups (*P*>0.05, Table 6). The levels of LAD and RAD were obviously higher in the SD group in comparison with those in the control group at 1 year after operation (*P*<0.05). A peak, SRa, and the use of statin were markedly lower in SD group when compared withose in the control group at 1 year after operation (*P*<0.05). There were no significant differences in E-peak, E/A value, S%, SRs, SRe, LAEF, LVEF, 6-min walk test, and ACEI/ARB medication between the two groups before operation and 1 year after operation (*P*>0.05). The incidence of non-arrhythmia palpitations failed to show statistical significance before operation and was higher in SD group compared with control after 1 year (*P*<0.05). The AF recurrence rate in SD group was higher than that in the control group (*P*<0.05). There were no statistical differences in the rate of rehospitalization and new stroke between the two groups (*P*>0.05) (Table 7).

The article "The influence of iatrogenic atrial septal defect on the prognosis of patients with atrial fibrillation between cryoablation and radiofrequency ablation" was published in 2020. Journal: Biosci Rep.

**Table 6:** Indexes comparison between SD and non-SD patients

Index	3 months		*P*-value	1 year		*P*-value
	ISD	Non-ISDN		ISD	Non-ISD	
LAD	37.97 ± 3.03	36.55 ± 4.64	0.093	37.44 ± 4.55	35.21 ± 3.21	<0.001
RAD	34.88 ± 3.89	35.88 ± 3.75	0.157	35.19 ± 2.80	34.12 ± 2.61	0.031
E peak	75.97 ± 21.16	70.88 ± 19.15	0.162	78.06 ± 18.09	77.23 ± 17.73	0.797
A peak	68.76 ± 18.79	70.64 ± 14.79	0.51	67.17 ± 11.73	72.96 ± 18.29	0.016
E/A peak	1.27 ± 0.45	1.13 ± 0.41	0.072	1.21 ± 0.37	1.10 ± 0.32	0.07
S%	29.84 ± 13.86	29.06 ± 11.96	0.733	37.56 ± 10.91	33.99 ± 9.82	0.056
SRs	1.56 ± 0.61	1.55 ± 0.52	0.92	1.85 ± 0.42	1.74 ± 0.44	0.181
SRe	−2.02 ± 0.74	−1.83 ± 0.75	0.177	−1.98 ± 0.84	−1.83 ± 0.69	0.259
SRa	−2.45 ± 0.70	−2.29 ± 0.68	0.366	−2.14 ± 0.69	−2.45 ± 0.69	0.047
LAEF	44.28 ± 13.47	45.61 ± 15.06	0.634	48.47 ± 16.68	53.63 ± 14.23	0.059
LVEF	59.08 ± 8.90	61.75 ± 7.67	0.069	64.66 ± 5.41	66.39 ± 5.46	0.075
6MWT	657.89 ± 100.42	668.52 ± 98.77	0.567	642.37 ± 120.84	678.55 ± 99.23	0.059
Non-arrhythmia palpitations (*n*)	11	63	0.208	12	57	0.049
Statin (*n*)	11	123	0.178	9	129	0.023
ACEI/ARB (*n*)	8	96	0.128	7	102	0.057
Rehospitalization (*n*)	–	–	–	6	32	0.302
New stroke (*n*)	–	–	–	1	3	0.363
AF recurrence (*n*)	–	–	–	15	77	0.046

**Table 7:** SD and non-SD AF recurrent rate comparison at 1 year after operation

Index	CB		*P*-value	RF		*P*-value
	IASD	Non-IASD		IASD	Non-IASD	
Recurrence	11 (22)	33 (119)	0.038	6 (10)	42 (142)	0.045

### Logistic regression analysis of SD

The logistic regression analysis showed that the use of statin (OR = 0.374, *P*=0.028) and the application of ACEI/ARB (OR = 0.347, *P*=0.031) were protective factors, whereas hypertension (OR = 2.606, *P*=0.039), LAD (OR = 1.133, *P*=0.014), left atrial operation time (OR = 1.016, *P*=0.041), and surgical plan (OR = 6.111, *P*=0.001) were risk factors for IASD. Hypertension and surgical procedures were independent risk factors.

## Discussion

Since the introduction of PVI for AF treatment in the 1990s, intervention of the left atrium through the right atrial septum is an essential pathway for this procedure. However, the iatrogenic atrial septal defect (IASD) caused by the interatrial septum did not attract attention. In recent years, with the advancement of technology and equipment, the intervention of left atrial surgery has been gradually increased. In addition to AF treatment, it was also applied in left atrial appendage and mitral valve repair. These surgical interspersing devices are larger and more complex, leading to the persistence of iASD and the presence of symptoms [10,11]. Numerous studies confirmed that the IASD caused by AF ablation was much higher than our estimate [12–15]. It was found that foramen ovale defects increased the risk of advanced arrhythmias and embolism, and the closure of the foramen ovale can reduce these risks [16]. However, for iASD treatment, current evidence supports the blockade of symptomatic IASD, including worsening heart failure, refractory hypoxemia, cryptogenic stroke, other embolism [17]. Prophylactic IASD closure is controversial in all iASD patients after intervention, and this treatment regimen has not been supported [18]. At present, there are few studies on whether IASD needs treatment after AF and its influence on long-term prognosis.

The article "The influence of iatrogenic atrial septal defect on the prognosis of patients with atrial fibrillation between cryoablation and radiofrequency ablation" was published in 2020. Journal: Biosci Rep.

All patients underwent standard PVI, and success rate was 100% immediately after surgery. At the postoperative follow-up, most of the atrial septal puncture sites had healed. The incidences of atrial SD were 24.11 and 15.60% in the cryoablation group at 3 months and 1 year, respectively. This result was lower than 20% IASD incidence reported by Sieira [19], which may be related to the fact that there were more patients in the cryoablation group and the use of second-generation balloon operation in our study. The incidences of atrial SD in radiofrequency ablation were 11.84 and 6.58% at 3 months and 1 years, respectively, which was similar to the results reported by Anselmino et al. [20]. In our trial, the incidence of IASD in the cryoablation group was significantly higher than that in the radiofrequency ablation group. During follow-up, no right-to-left shunt occurred in all patients with atrial SD. The high incidence of IASD in the cryoablation group may be related to the large diameter of the cryoplasty. The HR-CRP, TNI, and CKMB in the cryoablation group were significantly higher than those in the radiofrequency ablation group, which may be related to longer contact time and larger contact area between the balloon and the myocardial tissue during the ablation, resulting in more severe damage [21]. It may also be the cause of IASD in the frozen group. The level of LAD was higher, while SRe was lower in cryoablation group than those in the radiofrequency ablation group at 1 year after operation. The level of SRa in the cryoablation group was markedly lower than that in the radiofrequency ablation group at both 3 months and 1 year. LAEF showed no statistical difference at 1 year but it was lower in the cryoablation group than the radiofrequency ablation group after 3 months. The recurrence rate of AF in patients with IASD was significantly higher than that in patients without IASD (53.13 vs. 28.74%, *P*<0.05). Subgroup analysis revealed that the recurrence rate of AF was obviously higher in IASD patients than that in patients without IASD in cryoablation group at 1 year (50.00 vs. 27.73%, *P*<0.05). The recurrence rate of AF in patients with IASD was apparently higher than that in patients without IASD in the radiofrequency ablation group (60.00 vs. 29.58%, *P*<0.05), suggesting that IASD may increase the risk of postoperative AF recurrence. Controlling IASD may reduce postoperative AF recurrence and improve the success rate of surgery.

The article "The influence of iatrogenic atrial septal defect on the prognosis of patients with atrial fibrillation between cryoablation and radiofrequency ablation" was published in 2020. Journal: Biosci Rep.

The levels of LAD and RAD were obviously higher in SD group when compared with the control group at 1 year after operation, indicating that residual SD can lead to left and right atrial remodeling. At 1 year after operation, the A peak in the residual SD group was lower than that in the normal group, revealing that SD may decrease the effective ejection in the atrial systole. At 1 year after operation, the level of SRa in the residual SD group was lower than that in the control group. SD affected the atrial systolic response rate and the left atrial function. The incidence of non-arrhythmia palpitations was higher in residual SD group than that in the normal group at 1 year after surgery. Patients with atrial SD were more prone to appear discomfort symptom. The use of statin was lower, whereas the recurrence rate was higher in SD group than that in the control group. There were no significant differences in the 6-min walk test, new stroke, and rehospitalization rate between the two groups. It was found that residual SD can cause atrial remodeling, affect left atrial function, be more prone to non-arrhythmia-related palpitations, and have a higher AF recurrence rate. However, SD had no significant effects on cardiac function, exercise tolerance, rehospitalization rate, and new stroke.

There are still some limitations in the present study. For example, our results suggested that while there was no significant difference in baseline, there were younger patients and fewer patients with hypertension in the RF group that was associated with decreased SD. As hypertension was a significant independent risk factor, it may have some bearing on the result. In future research, we will design experimental schemes more rigorously.

The article "The influence of iatrogenic atrial septal defect on the prognosis of patients with atrial fibrillation between cryoablation and radiofrequency ablation" was published in 2020. Journal: Biosci Rep.

Binary logistic analysis of the potential influencing factors of IASD showed that the application of statins and ACEI/ARB were protective factors, while hypertension, LAD, left atrial operation time, and surgical plan were risk factors for IASD. Hypertension and surgical procedure were independent risk factors.

## Conclusion

Cryoablation showed significantly greater atrial injury than radiofrequency ablation, which was more likely to cause atrial remodeling and affect left atrial function. The SD incidence was obviously higher in cryoablation group than that in the radiofrequency ablation group. SD affected left atrial function and increased the risk of AF recurrence. Patients were more prone to some discomfort but it exhibited no significant impacts on exercise tolerance, stroke, and hospitalization. Hypertension, LAD, and left atrial operation time were risk factors for SD, whereas statin and ACEI/ARB drugs can reduce SD. Preoperative blood pressure control, surgical selection, and early intervention with statin and ACEI/ARB for patients with high-risk IASD should be considered.

## Abbreviations

ACEI: angiotensin-converting enzyme inhibitor
AF: atrial fibrillation
ARB: angiotensin receptor blocker
BMI: body mass index
BNP: B-type natriuretic peptide
CKMB: Creatine kinase-MB/Creatine kinase isoenzymes
CT: computed tomography
HR-CRP: HR-C-reactive protein
IASD: iatrogenic atrial septal defect
LAD: left atrial diameter
LAEF: left atrial ejection fraction
PVI: pulmonary vein isolation
RAD: right atrial diameter
SD: septal defect
SR: strain rate
SRa: left atrial systole
SRe: left ventricular diastolic
SRs: left ventricular systolic
TNI: Troponin I
